The article "Study of Hospitalization Costs in Patients with Cerebral Ischemia Based on E-CHAID Algorithm" was published in 2022. Journal: J Healthc Eng.

# Study of Hospitalization Costs in Patients with Cerebral Ischemia Based on E-CHAID Algorithm

**DOI:** 10.1155/2022/3978577

**Published:** 2022-05-02

**Authors:** Jing Gong, Ying Wang, Siou-Tang Huang, Herng-Chia Chiu

**Affiliations:** ^1^Institute for Hospital Management, Tsinghua University, Shenzhen, Guangdong, China; ^2^Department of Medical Administration, West China Hospital, Sichuan University, Chengdu, Sichuan, China; ^3^School of Public Health, Johns Hopkins University, Baltimore, USA; ^4^Department of Health Care Management and Medical Informatics, Kaohsiung Medical University, Kaohsiung, Taiwan

## Abstract

**Background:**

The aging of the population has led to a rapid increase in the prevalence of most neurological diseases between 1990 and 2016, with a growth rate of up to 117%, which has put enormous pressure on medical insurance funds. As one of the core diseases of disease diagnosis grouping, the hospitalization cost composition and grouping research of patients with cerebral ischemic disease can help to determine scientific payment standards and reduce the economic burden of patients.

**Aim:**

We aimed to understand the cost composition and influencing factors of hospitalized patients with cerebral ischemic diseases and to identify a reasonable cost grouping scheme.

**Methods:**

The data come from the homepage of medical records of inpatients with cerebral ischemia in a tertiary hospital in Sichuan Province from 2018 to 2020. After cleaning the data, a total of 5,204 pieces of data were obtained. Nonparametric tests and gamma regression models were used to explore the influencing factors of hospitalization costs. Taking the influencing factors as the predictor variables and the hospitalization cost as the target variable, the exhaustive Chi-squared automatic interaction detector (E-CHAID) algorithm was used to form the costs grouping, and the payment standard of the hospitalization cost for each group was determined. The rationality of cost grouping was evaluated by coefficient of variation (CV) and Kruskal–Wallis *H* test.

**Results:**

From 2018 to 2020, the average hospital stay of 5,204 inpatients with cerebral ischemic disease was 10.70 days, and the average hospitalization cost was 17,206.09 RMB yuan. Among the hospitalization costs, diagnosis costs and drug costs accounted for the highest proportion, accounting for 41.18% and 22.38%, respectively, in 2020. Gender, age, admission route, comorbidities and complications, super length of stay (>30 days), and discharge mode had significant effects on hospitalization costs (*P* < 0.05). Patients were divided into 10 cost groups, and the grouping nodes included comorbidities and complications, discharge mode, age, gender, and admission route. The CV of 9 of the 10 cost groups is less than or equal to 1. The Kruskal–Wallis *H* test showed that the difference between groups was statistically significant (*P* < 0.05).

**Conclusion:**

The cost grouping of patients with cerebral ischemic diseases based on the E-CHAID algorithm is reasonable. This study examined the effects of super length of stay (>30 days), comorbidities and complications, and age on hospitalization cost in patients with cerebral ischemic disease. This study can provide a theoretical basis for advancing the China Healthcare Security Diagnosis Related Groups (CHS-DRG) grouping program and medical expense payment, thereby reducing the disease burden of patients.

## 1. Introduction

Cerebral ischemic disease is brain tissue damage caused by vascular obstruction, including neuronal cell death and cerebral infarction, mainly manifested as ischemic stroke [1]. A survey of about 480,000 people in China showed that the prevalence and mortality of cerebral ischemia were 1114.8 and 114.8 per 100,000 people, respectively [2]. Studies have shown that the proportion of people discharged with neurological diseases in general hospitals in China is close to 11% [3], and cerebrovascular disease has become the leading cause of death among Chinese residents. Ischemic cerebrovascular disease accounts for 87% of new or recurring cerebrovascular diseases each year, and cerebral ischemic disease is also the fifth leading cause of death and disability in the United States [4].

In 2021, WHO released the Cross-departmental Global Action Plan for Epilepsy and Other Neurological Disorders [5], requiring countries to develop sustainable interventions for the prevention and management of neurological diseases based on local best practices, to ensure that patients with neurological diseases receive timely, affordable, and high-quality service. Patient hospital length of stay is one the most direct embodiment on efficiency as well as bed turnover rate, which consequently enhance patient access to service [6]. Hospitals have been using clinical management, such as the organizational structure, discharge planning, clinical pathway to shorten hospital length of stay, and reduce the medical cost [7]. DRG is believed to have a positive impact in optimizing hospital management, shortening the day of hospitalization. The appropriate bed management is not only to control medical cost, indirectly but also to reduce the financial burden for patients and third-party payers. Therefore, DRG is widely used among many medical systems as payment methods to achieve the objectives.

The reform of medical insurance payment includes two aspects: cost grouping and cost payment. The growing elderly population puts more and more pressure on the medical insurance fund pool [8, 9], so the reform of medical insurance payment methods will be the focus of long-term research in the future. According to the United Nations definition, China has entered an aging society at the beginning of the twenty-first century, and the proportion of the elderly population in China is expected to exceed 30% by 2050 [10].

Reasonable cost grouping is the premise of scientific cost payment. Based on BJ-DRG, CN-DRG, CR-DRG, and C-DRG, which are the most widely used and authoritative in China, CHS-DRG grouping program [11] was formulated and released by the National Healthcare Security Administration in 2019. CHS-DRG mainly uses the national health insurance code, including “Medical security disease diagnosis classification and code (ICD-10)” and “Medical security surgery classification and code (ICD-9-CM-3).” As one of the 376 adjacent diagnosis related groups (ADRG) in the CHS-DRG grouping scheme, the cerebral ischemic disease group has research value.

Due to the skewed distribution of hospitalization cost, it is usually necessary to logarithmically transform it to use multiple linear regression [12]. Although Logistic regression models do not require data distribution, cost data integrity after classification is reduced [13]. Gamma regression model is a type of generalized linear model that can process data through logarithmic links to reduce data loss and ensure data integrity [14], so it is gradually applied to medical cost analysis [15, 16].

There have been previous studies on hospitalization cost [17–19], but not many studies on cerebral ischemic diseases. Based on the newly released CHS-DRG grouping scheme in China, we firstly calculated the CV of cerebral ischemic diseases ADRG group, which is the premise of cost grouping. Then we analyze the composition, influencing factors, and cost grouping of cerebral ischemic disease patients, and finally tries to determine the cost standard of each cost grouping, so as to reduce the disease burden and economic pressure of patients.

## 2. Material and Methods

### 2.1. Setting

This study is a single-center retrospective study with data from a large tertiary hospital in Sichuan Province, China. The medical center has more than 4,000 acute care beds. In 2021, the hospital has 7.75 million outpatient visits (included emergency), and more than 283,000 admissions, with an average length of stay of 6.80 days. The hospital has been among the best for many years which can represent the medical level of China's general acute hospital and has certain reference significance for other countries in the world.

### 2.2. Data Source and Processing

The data come from the information system of a tertiary hospital in Sichuan Province, including the basic information and cost data of patients with cerebral ischemic diseases. In the CHS-DRG grouping scheme (Figure 1), patients with cerebral ischemic disease were divided into the BR2 ADRG group, and no DRG group subdivision was performed. A total of 6214 cases of inpatients with cerebral ischemic diseases from 2018 to 2020 were collected, and 5204 cases remained after data processing. Data exclusion criteria: (1) cases with blank/missing items; (2) cases in which the major diagnosis or major operation code is not included in the CHS-DRG grouping scheme; (3) cases in which the length of stay is longer than 60 days; (4) cases in which hospitalization cost are less than 1 percentile or more than 99 percentiles.

According to the MCC&CC inclusion and exclusion tables in the CHS-DRG grouping scheme, we sorted out the comorbidities and complications of patients with cerebral ischemic diseases. If a patient had any secondary diagnosis on the MCC&CC inclusion table and the primary diagnosis was not on the exclusion table, the case had MCC or CC. The comorbidities and complications of the patients were divided into three groups, the first group had major comorbidities and complications (MCC), the second group had comorbidities and complications (CC), and the third group had no comorbidities and complications (Non-CC).

### 2.3. Classification and Description of Hospitalization Expenses

The classification of the total hospitalization cost is based on the homepage of Chinese hospitals [20], of which the diagnosis cost and drug cost account for the highest proportion. Diagnosis cost items include pathological diagnosis, laboratory diagnosis, imaging diagnosis, and clinical diagnosis. Drug cost includes cost items in western medicine, Chinese patent medicine, and Chinese herbal medicine. Comprehensive medical service cost includes cost items of physician fee, nursing care, bed, and others.

### 2.4. Statistical Analysis

Because the hospitalization cost does not conform to the normal distribution, the nonparametric test was used to carry out univariate analysis of the hospitalization cost, and the Gamma regression model was used to carry out the multivariate analysis of the hospitalization cost and calculate the cost ratio (CR). In univariate analysis, the Mann–Whitney *U* test was used for cost comparisons between two groups of variables, and the Kruskal–Wallis *H* test was used for cost comparisons among multiple groups. Taking the hospitalization cost as the dependent variable, and the factors that have a high degree of influence on the hospitalization cost as the grouping node, the E-CHAID algorithm is used to group the cost. CV [21] and Kruskal–Wallis *H* test [22] were used to evaluate the reasonableness of cost grouping. Excel 2019 software was used for data entry and SPSS 26.0 and SPSS Modeler 18.0 were used for statistical analysis.

## 3. Results

### 3.1. The Premise of Cost Grouping

The document shows [23] that ADRG group with CV greater than 1 can be subdivided, and the CV of hospitalization cost in the cerebral ischemic disease ADRG group is calculated to be 1.18. The cost grouping process of this study is shown in Figure 2.

### 3.2. General Information

From 2018 to 2020, there were 5204 patients in the cerebral ischemia disease ADRG group, including 3215 male patients (61.78%) and 1989 female patients (38.22%). The age of the patients ranged from 0 to 99 years old, with an average age of 65.30 years. The length of hospital stay ranged from 1 to 60 days, with an average hospital stay of 10.70 days.

### 3.3. Composition of Inpatient Hospitalization Expenditure

As shown in Table 1, the total hospitalization cost of the cerebral ischemic disease ADRG group from 2018 to 2020 was 89.54 million RMB yuan, and the average hospitalization cost was 17,206.09 RMB yuan, of which the diagnosis cost and drug cost accounted for the highest proportion, accounting for 41.18% and 22.38%, respectively, in 2020. In the past three years, the proportion of comprehensive medical service cost has decreased year by year, and the proportion of treatment cost, and blood and blood products cost has increased year by year.

### 3.4. Factors Affecting Inpatient Hospitalization Expenditure

#### 3.4.1. Univariate Analysis

As shown in Table 2, in addition to allergy, gender, age, social insurance, admission route, comorbidities and complications, discharge mode, and super length of stay (>30 days) have statistically significant effects on hospitalization cost (*P* < 0.05).

#### 3.4.2. Multivariate Analysis Using Gamma Model

Results (Table 3) showed that gender, age, comorbidities and complications, admission route, super length of stay (>30 days), and discharge mode all had an impact on hospitalization cost. Through the cost ratio, it can be seen that the super length of stay (>30 days), age, and comorbidities and complications have a greater impact on the hospitalization cost. Compared with patients whose hospitalization days were less than or equal to 30 days, patients with super length of stay (>30 days) spent more medical costs (CR = 4.23); compared with patients aged 0–17 years old, patients older than 65 years old spent more medical costs (CR = 2.63).

### 3.5. Grouping and Verification of Inpatient Hospitalization Cost

Since the length of hospital stay in China is affected by many factors, and there are large disparities between different hospitals, the super length of stay (>30 days) is not used as a grouping variable. Selecting the meaningful factors of multivariate analysis as grouping nodes, using CART and E-CHAID algorithms to construct cost groups, and form 2 and 10 cost groups respectively. As shown in Table 4, taking into account the number of groups and the mean absolute error, we finally chose the E-CHAID model for subsequent analysis.

As shown in Table 5, 5204 patients were divided into 10 cost groups, and the grouping nodes included comorbidities and complications, discharge mode, age, gender, and admission route. The fourth group had the largest number of patients with 1823 patients (35.03%), these patients had general comorbidities and complications, and were older than 65 years. The seventh group had the smallest number of patients, with only 56 patients (2.09%), who had no comorbidities and complications, were admitted through outpatient and other routes, and were younger than 18 years old. Among the 10 cost groups, the CV of nine groups are all less than or equal to 1, and the grouping is reasonable. The Kruskal–Wallis *H* test was performed on the cost groups, and the difference between the groups was statistically significant (*P* < 0.001).

### 3.6. Cost Payment Standard

As shown in Table 5, the median medical cost of each group is taken as the standard cost. The 75th percentile of cost per group plus 1.5 times the interquartile range was used as the upper limit of medical costs for that group, and cases above the upper limit were defined as excess amount [24, 25]. The second group (MCC, transferred to another hospital, death and others) had the highest standard cost, about 25,000 RMB yuan; the seventh group (Non-CC, outpatient and other admission, <18 years old) had the lowest standard cost, close to 1,500 RMB yuan. The fourth group (CC, ≤65 years old) had the highest excess rate at 10.43%, and the ninth group (Non-CC, outpatient and other admission, 18–65 years old, female) had the lowest excess rate at 0.56%.

## 4. Discussion

According to the CHS-DRG grouping scheme, the CV of the cerebral ischemic disease ADRG group is 1.18, and the patient's personal characteristics and disease characteristics have a certain influence on the hospitalization cost, so it is reasonable to group the cost for the ADRG group. At the same time, it also shows that the applicability of the grouping scheme of CHS-DRG needs to be improved.

The prevalence of most neurological diseases increased rapidly from 1990 to 2016, with a growth rate of 117% due to an aging population [26]. As a common neurological disease, cerebral ischemic disease has the characteristics of high mortality and high disability rate [5], which will cause a heavy economic and labor burden to patients, families, and society. The results of the study showed that from 2018 to 2020, the average length of hospital stay for patients with cerebral ischemic disease was 10.70 days, and the average hospitalization cost was 17,206.09 RMB yuan. Among the hospitalization cost, diagnosis cost and drug cost accounted for the highest proportion, accounting for 41.18% and 22.38% in 2020, respectively. Diagnosis of cerebral ischemic disease, selection of treatment options, and assessment of prognostic status involve imaging studies [27, 28], which may result in high diagnostic costs. The high proportion of diagnostic costs is in line with the trend of medical reform, and early diagnosis is of great significance for the prevention and treatment of cerebral ischemic diseases. The use of imported drugs (the thrombolytic agent alteplase (rt-PA) [29]) and the nonreimbursement of certain drugs by medical insurance are possible reasons for the high cost of drugs [30, 31]. The proportion of drug costs in the total cost in China is significantly higher than the international proportion [32, 33], so reducing the drug costs of patients with cerebral ischemic disease has positive significance for reducing the disease burden of such patients [34].

Age has important implications for patient classification in many countries [35, 36]. The research results show that the average age of patients with cerebral ischemia is 65.30 years old, and the hospitalization cost of patients over 65 years old is 2.63 times that of patients aged 0–17 years old, which is in line with the natural pathological characteristics of the disease. Meanwhile, the elderly tend to have more comorbidities and complications because of the decline of physical function and thus spend more medical expenses [36].

The homogeneity of patients in the DRG group is a prerequisite for reasonable reimbursement by medical insurance. In order to ensure the homogeneity of patients in each group, it is necessary to carefully select categorical variables [37]. Through the cost ratio, it can be found that super length of stay (>30 days), comorbidities and complications, and discharge mode have a greater impact on hospitalization cost. The hospitalization cost of patients with super length of stay (>30 days) is significantly higher than that of patients with hospitalization days less than or equal to 30 days (CR = 4.23), which requires hospitals to follow evidence-based guidelines, strengthen clinical pathway management, and standardize similar patients' treatments and costs, thereby reducing the disease and economic burden of individual patients. Comorbidities and complications are important influencing factors in hospitalization costs. It can be seen from the grouping results that the standard cost of the second group (MCC, transferred to another hospital, death and others) is the highest, about 25,000 RMB yuan, which may be related to the increased difficulty of treatment due to the higher severity of the patients included in this grouping [18]. Discharge mode is also influenced to some extent by the severity of the disease, for example, patients who are transferred to another hospital on advice or who die tend to have more severe disease.

Computational cost grouping usually includes three methods: CART, CHAID, and E-CHAID, of which E-CHAID is an improved method of CHAID [19]. We found that E-CHAID has smaller model error and higher grouping performance than CART, which is consistent with other research results [38]. The results of CV and Kruskal–Wallis *H* test show that the cost grouping in this study is reasonable, and the grouping scheme is meaningful, which can provide a feasible method for the medical insurance department to improve the disease grouping scheme and pay for diseases [39].

## 5. Conclusion

Based on the CHS-DRG grouping scheme, this study analyzed the composition and influencing factors of medical costs for inpatients with cerebral ischemic diseases, and used the E-CHAID algorithm to group costs. This study further verifies the applicability of the CHS-DRG grouping scheme and helps to optimize the DRG grouping system. This study also provides a theoretical basis for cost control of cerebral ischemic diseases, which is beneficial to reduce the economic burden of patients, and provides suggestions for other developing countries to improve the disease diagnosis grouping system.

### 5.1. Limitations of the Study

The advantage of this study lies in the rich sample size and the data from representative general hospitals. However, this study also has certain limitations. Due to the availability of data, the data in this study are only from one hospital, and multicenter studies need to be added in the future to make the findings more generalizable. In addition, the hospitalization cost measured in this article is only a part of the direct economic burden [39], so the actual cost of the patient may be higher.

## Figures and Tables

**Figure 1:** The grouping process of CHS-DRG grouping scheme.

**Figure 2:** The grouping process of sample patients with cerebral ischemia.

**Table 1:** Composition of hospitalization cost from 2018–2020 (*N* = 5204).

Year	2018 (*N* = 1892)		2019 (*N* = 1909)		2020 (*N* = 1403)	
Cost category (RMB yuan)	Mean cost	%	Mean cost	%	Mean cost	%
Diagnosis cost	7002.85	42.69	6944.94	39.86	7409.75	41.18
Drug cost	3762.32	22.93	4341.63	24.92	4026.44	22.38
Comprehensive medical service cost	2580.27	15.73	2514.80	14.43	2491.84	13.85
Rehabilitation cost	1065.62	6.50	988.00	5.67	1191.05	6.62
Consumables cost	780.23	4.76	746.37	4.28	909.14	5.05
Treatment cost	575.62	3.51	698.46	4.01	782.53	4.35
Blood and blood product cost	18.82	0.11	88.96	0.51	176.71	0.98
Other cost	619.28	3.77	1098.63	6.31	1005.46	5.59
Overall	16405.00		17421.78		17992.90	

**Table 2:** Univariate analysis of cerebral ischemic disease ADRG group (*N* = 5204).

Variable	Assignments	*N*	%	Rank mean in RMB yuan	Z/H/F	*P*
Sex	Male	3,215	61.78	2,645.55	−2.628	0.009
	Female	1,989	38.22	2,532.91		
Age	1–17	68	1.31	677.17	288.525	<0.001
	18–65	2,271	43.64	2,316.16		
	>65	2,865	55.05	2,875.17		
Allergic	No	2,672	51.35	2,606.35	−0.190	0.849
	Yes	2,532	48.65	2,598.44		
Social insurance	No	4599	88.37	2,602.05	41.131	<0.001
	Yes	605	11.63	2,433.93		
Comorbidities and complications	MCC	1,167	22.43	3,431.38	838.131	<0.001
	CC	3,002	57.69	2,633.63		
	Non-CC	1,035	19.89	1,577.61		
Admission route	Emergency	2,853	54.82	2,836.93	−12.400	<0.001
	Outpatient and others	2,351	45.18	2,318.01		
Discharge mode	Discharged home	5,030	96.66	2,561.76	121.377	<0.001
	Transferred to another hospital	63	1.21	3,880.44		
	Death	91	1.75	3,938.09		
	Others	20	0.38	2,746.35		
LOS >30 days	No	4,991	95.91	2,503.22	−23.076	<0.001
	Yes	213	4.09	4,928.87		
LOS (Mean ± SD)		10.70 **±** 8.61			106.688	<0.001

**Table 3:** Multivariate analysis of cerebral ischemic disease ADRG group (*N* = 5204).

Variables	Assignments	Marginal mean in RMB yuan	Marginal mean's difference in RMB yuan	Cost ratio	95% CI		*P*
Sex	Ref: female	27496.58					
	Male	28940.61	1444.04	1.05	1.02	1.09	0.004
Age	Ref:0–17	15666.35					
	18–65	34761.31	19094.96	2.22	1.91	2.58	<0.001
	>65	41220.71	25554.36	2.63	2.27	3.06	<0.001
Social insurance	Ref: yes	27604.41					
	No	28827.55	1223.14	1.04	0.99	1.10	0.108
Admission route	Ref: outpatient and others	25710.88					
	Emergency	30950.62	5239.73	1.20	1.16	1.25	<0.001
Comorbidities and complications	Ref: non-CC	18895.52					
	CC	27889.88	8994.36	1.48	1.41	1.54	<0.001
	MCC	42596.49	23700.97	2.25	2.14	2.38	<0.001
LOS >30 days	Ref: no	13711.32					
	Yes	58037.29	44325.97	4.23	3.89	4.61	<0.001
Discharge mode	Ref: discharged home	20378.89					
	Transferred to another hospital	35905.05	15526.16	1.76	1.51	2.05	<0.001
	Death	31563.01	11184.12	1.55	1.36	1.76	<0.001
	Others	27419.41	7040.52	1.35	1.03	1.76	0.031

**Table 4:** Comparison of CART and E-CHAID models (*N* = 5204).

Model	Linear correlation	Mean absolute error	Standard deviation	Number of groups
CART	0.309	10426.817	19296.419	2
E-CHAID	0.352	10209.751	18985.752	10

**Table 5:** Grouping results and the predicted medical costs (*N* = 5204).

Group number	Classification description	*N*	CV	Median in RMB yuan	IQR	P75	Upper limit	Excess amount *N* (%)
1	MCC, discharged home	1046	1.13	16861.55	20478.52	30826.32	61544.09	107 (10.23)
2	MCC, transferred to another hospital, death and others	121	1.11	24554.26	32125.81	46340.91	94529.62	11 (9.09)
3	CC, ≤65 years old	1179	0.84	10527.18	6991.76	14977.50	25465.14	123 (10.43)
4	CC, >65 years old	1823	0.92	11928.30	8956.58	17892.89	31327.76	177 (9.71)
5	Non-CC, emergency admission, male	269	0.60	9875.89	5329.05	13127.80	21121.38	20 (7.43)
6	Non-CC, emergency admission, female	169	0.45	9414.20	4938.46	12336.98	19744.67	8 (4.73)
7	Non-CC, outpatient and other admission, <18 years old	56	2.09	1484.30	51.62	1527.48	1604.91	11 (19.64)
8	Non-CC, outpatient and other admission, 18–65 years old, male	212	0.94	6811.34	8170.03	9705.90	21960.94	11 (5.19)
9	Non-CC, outpatient and other admission, 18–65 years old; female	179	0.74	5584.74	6597.86	8098.58	17995.37	1 (0.56)
10	Non-CC, outpatient and other admission, >65 years old	150	0.66	8502.10	4613.23	11123.75	18043.59	15 (10.00)

## Data Availability

The data come from the homepage of medical records of inpatients with cerebral ischemia in a tertiary hospital in Sichuan Province, and the use of the data need to obtain approval from the relevant departments of the hospital.
